RETRACTED

# A Posterior TAP Block Provides More Effective Analgesia Than a Lateral TAP Block in Patients Undergoing Laparoscopic Gynecologic Surgery: A Retrospective Study

**DOI:** 10.1155/2016/4598583

**Published:** 2016-01-28

**Authors:** Sakatoshi Yoshiyama, Hironobu Ueshima, Ryomi Sakai, Hiroshi Otake

**Affiliations:** Department of Anesthesiology, Showa University Hospital, 1-5-8 Hatanodai, Shinagawa-ku, Tokyo, 142-8666, Japan

## Abstract

*Background*. There are a few papers that compared the lateral transversus abdominis plane (TAP) block with the posterior TAP block. Our study aimed to compare retrospectively the quality of analgesia after laparoscopic gynecologic surgery using the lateral TAP block with general anesthesia versus the posterior TAP block with general anesthesia.* Method*. Sixty-seven adult female patients were included in this retrospective study. Of these patients, thirty-four patients received the lateral TAP block with general anesthesia (lat. TAP group), and the rest of thirty-three patients received the posterior TAP block with general anesthesia (pos. TAP group). Pain scores both at rest and at movement and the use of additional analgesic drugs were recorded in the postoperative care unit within twenty-four hours after the operation. Postoperative complications were noted.* Results*. Patients who received pos. TAP reported lower visual analog scale (VAS) pain scores in all points, within twenty-four hours after the operation, than patients who received lat. TAP. Moreover, with the use of additional analgesic drugs, the incidence of nausea and vomiting during the first twenty-four hours after surgery was lower in the pos. TAP group than in the lat. TAP group.* Conclusion*. The posterior TAP block provided more effective analgesia than the lateral TAP block in patients undergoing laparoscopic gynecologic surgery.

## 1. Introduction

Laparoscopic surgery has been increasingly performed in recent years. Intravenous morphine has been used as one of the postoperative analgesia drugs for these laparoscopic surgeries, but morphine causes complications such as respiratory depression and circulatory depression [1]. Therefore, people from old times have hesitated to use morphine as postoperative analgesia [2].

Since the publishing of a paper on the transversus abdominis plane (TAP) block in two thousand and one [3, 4], the TAP block has been used as an analgesia for somatic pain in lower abdominal surgeries and has decreased the amount of morphine used [5–7]. There are two major types of the TAP block, the lateral approach and the posterior approach. However, there are a few papers that compared the lateral TAP block with the posterior TAP block [8]. The posterior TAP block is said to reduce postoperative morphine [8], but the analgesia of the posterior TAP block in postoperative period has not been well known. Therefore, the differences in efficacy between the lateral TAP block and the posterior TAP block also are still unclear. In this study, we compared the analgesia efficacy of the posterior TAP block with the lateral TAP block for the laparoscopic gynecologic surgery retrospectively.

RETRACTED

## 2. Materials and Methods

This retrospective study was approved by the Showa University Hospital Institutional Review Board (approval number 1895). In addition, the study was registered at the University Hospital Medical Information Network (UMIN ID number 000019314). In this study, we investigated female patients who had laparoscopic gynecologic surgery at Showa University Hospital from April, two thousand and fifteen, to September, two thousand and fifteen. Exclusion criteria were the conversion from laparoscopic surgery to open surgery and secondary surgery.

Perioperative data of the subjected patients were collected retrospectively, including age, height, weight, American Society of Anesthesiologists (ASA) classification, operation time, anesthesia time, surgery contents, visual analog scale (VAS) pain scores and the number of additional analgesic drugs used, and the complications (i.e., nausea and vomiting) within twenty-four hours after the operation. VAS pain scores were measured at one, two, six, twelve, and twenty-four postoperative hours during rest and at twelve and twenty-four postoperative hours during movement of sitting up in bed. The researchers were two nurses. They were used to measure the VAS. In my hospital, all patients move to the intensive care unit (ICU) after laparoscopic gynecologic surgery. Each patient who performed laparoscopic gynecologic surgery moved regularly to the ICU measures at one, second, six, twelve, and twenty-four postoperative hours during rest and at twelve and twenty-four postoperative hours during movement by nurses being in the ICU. The additional analgesic drug was fifteen mg of intravenous pentazocine when the patient complained about pain. The frequency of complications such as nausea and vomiting were counted as the number of patients injected with ten mg of intravenous metoclopramide. We compared those data between two groups of patients, who received the lateral TAP block with general anesthesia and the posterior TAP block with general anesthesia.

The lateral TAP block: forty mL of 0.375% levobupivacaine (20 mL into each side) was injected in the TAP to the lateral abdominal wall in the midaxillary line, between the lower costal margin and iliac crest [8].

RETRACTED

The posterior TAP block: forty mL of 0.375% levobupivacaine (20 mL into each side) was injected in the TAP in the area of the triangle of Petit [8].

Each anesthesiologist decides on the type of the TAP block by himself or herself. There have been no rules on how the type of the TAP block is decided upon, but anesthetic record has been written. The volume and concentration of TAP block are decided for all cases.

Statistical analysis was performed utilizing JMP® 11 (SAS Institute Inc., Cary, NC, USA). Patient demographics, VAS pain scores, the number of additional analgesic drugs injected, and the frequency of complications were analyzed by using the Mann-Whitney *U* test, Student's *t*-test, and *χ* ^2^ test, retrospectively. Data of age, height, weight, operation time, anesthesia time, and VAS pain score were expressed as a median (twenty-fifth to seventy-fifth percentiles) (cm), number of additional analgesic drugs injected expressed as average (standard deviation), and the intravenous metoclopramide expressed as frequency with percentages (%), and we used Fisher's exact test. The level of significance for both tests was set at *P* < 0.05.

## 3. Results

During the study period, seventy-three patients underwent laparoscopic gynecologic surgery. Of these patients, thirty-four patients received the lateral TAP block under general anesthesia (lat. TAP group) and thirty-three patients received the posterior TAP block under general anesthesia (pos. TAP group). Six patients (two patients in lat. TAP group and four patients in pos. TAP group) were excluded from the study because of the criteria.  Table 1 is the comparison of patient's demographics, ASA classification, operation time, and anesthesia time. Surgery contents were shown in Table 2. VAS pain scores of lat. TAP group at one, two, six, twelve, and twenty-four postoperative hours during rest were 3.0 (3–4.5), 4.0 (3.5–5), 4.5 (4–6), 3.5 (3-4), and 3.0 (3-4), respectively, while those of pos. TAP group at one, two, six, twelve, and twenty-four postoperative hours during rest were 2.0 (1.5–2), 2.0 (1.5–2.5), 2.8 (2–3.5), 2.0 (1-2), and 2.0 (1-2), respectively (Table 3, Figure 1). As shown in Table 3, VAS pain scores of pos. TAP group were significantly lower than those of lat. TAP group in all test periods. VAS pain scores of lat. TAP group at twelve and twenty-four postoperative hours during movement were 3.0 (3-4) and 5.0 (4–7), while those of pos. TAP group at twelve and twenty-four postoperative hours during movement were 2.0 (1-2) and 3.0 (2.5–3.5) (Figure 2). As compared with those of lat. TAP group, VAS pain scores of pos. TAP group scores were significantly lower in both time periods (Table 3). The amounts of additional pentazocine in pos. TAP group (1.4 (0.5)) were significantly lower than those in lat. TAP group (3.0 (1.1)). Metoclopramide was injected for 17.6% patients in lat. TAP group, and for 6.1% patients in pos. TAP group, and the difference was significant (Table 4).

RETRACTED

## 4. Discussion

This study suggests that the posterior TAP block could provide better analgesia than the lateral TAP block for laparoscopic gynecologic surgery in perioperative period. Better analgesia enabled us to decrease the incidence of complications and the usage of additional analgesics.

For the TAP block, reported by Rafi et al, injecting local anesthetic in the lumbar triangle of Petit can provide better postoperative analgesia in lower abdominal surgery [3]. Rafi's technique of TAP block was a landmark technique, which has the risk of complications such as organ injury, mistaken puncture of superficial circumflex iliac perforator, and nerve injury which were pointed out [9, 10]. The breakthrough in the technique happened when the ultrasound-guided TAP block was reported by Manatakis et al., which could predict improving patient's security [11]. However, the efficacy of the TAP block performed by the ultrasound-guided technique was ineffective because an injection site may not have been the lumbar triangle of Petit [12, 13]. The new approach called the posterior TAP block was introduced to improve the efficacy. On the other hand, the previous approach was called the lateral TAP block. The injection site of the posterior TAP block is almost the same as that of the TAP block reported by Rafi. This study showed that the posterior TAP block is an effective analgesia for lower abdominal surgery.

The prime cause of postoperative pain for laparoscopic gynecologic surgery is said to derive from the visceral pain in the uterus and the vagina. The posterior TAP block is believed to relieve the visceral pain and this theory is proved with the result of this study. Walter et al. reported that local anesthetic spread to the thoracic paravertebral space in the posterior TAP block [14]. The reach of local anesthetics into the thoracic paravertebral space may result in blocking the sympathetic nerve and relieving the visceral pain. The effective analgesia in perioperative period by the posterior TAP block enabled us to decrease the amounts of additional analgesia and the frequency of complications such as nausea and vomiting.

The injection site of the posterior TAP block in this study was the lumbar triangle of Petit, but several other approaches of the posterior TAP blocks including quadratus lumborum blockade have been reported in recent years [15, 16]. The difference among these posterior TAP blocks is still not known in detail, which needs further investigations.

RETRACTED

There were some limitations of this study. VAS scores were affected by additional analgesic drug. If a patient required additional analgesic drug at, say, 1 hour after surgery, then it would be expected to have an impact on the VAS score at the 2-hour time point. In the future, we must solve this problem. This study also was a retrospective study, not a randomized control study. We also do not know the appropriate volume and concentration for the TAP blocks. In this study, we focused only on the first 24 hours after surgery because the TAP block was not a continuous administration but a single shot. Some surgeries require analgesia longer than 24 hours. These problems are left for the future study.

In conclusion, we found that the posterior TAP block could provide more effective analgesia than the lateral TAP block in patients undergoing laparoscopic gynecologic surgery.

## Figures and Tables

**Figure 1:** Postoperative VAS scores at one, two, four, six, twelve, and twenty-four postoperative hours during rest: data expressed as a median (twenty-fifth to seventy-fifth percentiles).

**Figure 2:** Postoperative VAS scores twelve and twenty-four postoperative hours during movement: data expressed as a median (twenty-fifth to seventy-fifth percentiles).

**Table 1:** Patients demographics data: age, height, weight, operation time, and anesthesia time. Data except ASA classification expressed as median (twenty-fifth to seventy-fifth percentiles). ASA classification expressed the numbers.

	Lat. TAP group (*n* = 34)	Pos. TAP group (*n* = 33)	*P*
Age (years)	40 (35–45)	41 (36–27)	0.65
Height (cm)	159.5 (153.5–163)	158.5 (155–162.5)	0.74
Weight (kg)	56 (48–60)	52.5 (49–60.5)	0.81
ASA classification (I/II/III)	8/25/1	7/24/2	—
Operation time (minutes)	120 (80–170)	110 (75–185)	0.98
Anesthesia time (minutes)	160 (115–205)	150 (120–220)	0.98

**Table 2:** Surgery contents. *P* calculated by using Fisher's exact test.

	Lat. TAP group (*n* = 34)	Pos. TAP group (*n* = 33)	*P*
Total hysterectomy	6	5	0.8
Uterine myomectomy	14	12	0.82
Oophorectomy	8	7	0.68
Tubectomy	5	8	0.37
The others	1	1	1.00

**Table 3:** Postoperative VAS scores during both rest and movement: data expressed as median (twenty-fifth to seventy-fifth percentiles).

	Lat. TAP group (*n* = 34)	Pos. TAP group (*n* = 33)	*P*
VAS at rest (h)			
1	3.0 (3.0–4.5)	2.0 (1.5–2.0)	<0.0001
2	4.0 (3.5–5.0)	2.0 (1.5–2.5)	<0.0001
6	4.5 (4.0–6.0)	2.5 (2.0–3.5)	<0.0001
12	3.5 (3.0–4.0)	2.0 (1.0–2.0)	<0.0001
24	3.0 (3.0–4.0)	2.0 (1.0–2.0)	<0.0001
VAS at movement (h)			
12	3.0 (3.0–4.0)	2.0 (1.0–2.0)	<0.0001
24	5.0 (4.0–7.0)	3.0 (2.5–3.5)	<0.0001

RETRACTED

**Table 4:** Postoperative dates except some VAS scores: data of the amounts of additional pentazocine expressed as average (standard deviation) and amounts of the intravenous metoclopramide expressed as frequency with percentages (%).

	Lat. TAP group (*n* = 34)	Pos. TAP group (*n* = 33)	*P*
The amounts of additional pentazocine 15 mg	3.0 (1.1)	1.4 (0.5)	<0.0001
The number of people who used intravenous metoclopramide 10 mg	17.6	6.1	0.02
